The article "Involvement of the JNK/FOXO3a/Bim Pathway in Neuronal Apoptosis after Hypoxic–Ischemic Brain Damage in Neonatal Rats" was retracted in 2020. Reasons: duplicated images; original data or images not available.

# Involvement of the JNK/FOXO3a/Bim Pathway in Neuronal Apoptosis after Hypoxic–Ischemic Brain Damage in Neonatal Rats

**DOI:** 10.1371/journal.pone.0132998

**Published:** 2015-07-14

**Authors:** Deyuan Li, Xihong Li, Jinlin Wu, Jinhui Li, Li Zhang, Tao Xiong, Jun Tang, Yi Qu, Dezhi Mu

**Affiliations:** 1 Department of Pediatrics, West China Second University Hospital, Sichuan University, Chengdu 610041, China; 2 Key Laboratory of Obstetric & Gynecologic and Pediatric Diseases and Birth Defects of Ministry of Education, Sichuan University, Chengdu, Sichuan 610041, PR China; 3 Department of Neurology, University of California San Francisco, San Francisco, CA 94143, United States of America; University of Modena and Reggio Emilia, ITALY

## Abstract

c-Jun N-terminal kinase (JNK) plays a key role in the regulation of neuronal apoptosis. Previous studies have revealed that forkhead transcription factor (FOXO3a) is a critical effector of JNK-mediated tumor suppression. However, it is not clear whether the JNK/FOXO3a pathway is involved in neuronal apoptosis in the developing rat brain after hypoxia-ischemia (HI). In this study, we generated an HI model using postnatal day 7 rats. Fluorescence immunolabeling and Western blot assays were used to detect the distribution and expression of total and phosphorylated JNK and FOXO3a and the pro-apoptotic proteins Bim and CC3. We found that JNK phosphorylation was accompanied by FOXO3a dephosphorylation, which induced FOXO3a translocation into the nucleus, resulting in the upregulation of levels of Bim and CC3 proteins. Furthermore, we found that JNK inhibition by AS601245, a specific JNK inhibitor, significantly increased FOXO3a phosphorylation, which attenuated FOXO3a translocation into the nucleus after HI. Moreover, JNK inhibition downregulated levels of Bim and CC3 proteins, attenuated neuronal apoptosis and reduced brain infarct volume in the developing rat brain. Our findings suggest that the JNK/FOXO3a/Bim pathway is involved in neuronal apoptosis in the developing rat brain after HI. Agents targeting JNK may offer promise for rescuing neurons from HI-induced damage.

## Introduction

c-Jun N-terminal kinase (JNK), a member of the mitogen-activated protein kinase (MAPK) family, has been shown to be activated in several models of neuronal apoptosis induced by excitotoxicity, trophic factor withdrawal and ischemia [1]. Inhibition of JNK signaling through genetic and pharmacological approaches protects neurons against several different apoptotic stimuli [2,3,4]. Although JNK has been established as a key player in neuronal apoptosis, the mechanisms that link JNK to neuronal apoptosis have not been clearly defined.

The article "Involvement of the JNK/FOXO3a/Bim Pathway in Neuronal Apoptosis after Hypoxic–Ischemic Brain Damage in Neonatal Rats" was retracted in 2020. Reasons: duplicated images; original data or images not available.

Mammalian forkhead transcription factor (FOXO) is a critical effector of JNK-mediated tumor inhibition [5,6]. The FOXO family consists of four members: FOXO1a; FOXO3a; FOXO4; and FOXO6 [5]. Among them, FOXO3a is closely related to cellular apoptosis, aging, proliferation, metabolism, differentiation and tumorigenesis [7,8,9,10]. FOXO3a activity is regulated at different levels, and its phosphorylation status plays a pivotal role in regulating its subcellular localization and transcriptional activities [11]. When FOXO3a is phosphorylated by protein kinase B (Akt), FOXO3a binds 14-3-3 protein and is retained in the cytoplasm. Conversely, FOXO3a dephosphorylation results in its translocation from the cytoplasm to the nucleus [12,13].

FOXO3a regulation involves multiple pathways, including the pro-survival PI3K/Akt pathway and the pro-apoptotic JNK pathway [9]. JNK regulates the activities of FOXO3a at different levels [14,15]. Activation of JNK in vitro leads to phosphorylation of 14-3-3 at serine 184, which in turn causes dissociation of FoxO3a from 14-3-3 in the cytoplasm, resulting in nuclear localization of FOXO3a [16]. This translocation induces FOXO3a target genes, such as the pro-apoptotic protein Bcl-2-interacting mediator of cell death (Bim). Bim has been shown an important mediator of neuronal death in neonatal hypoxia-ischemia models [17]. As a member of the Bcl-2 family, Bim activation can directly interact with pro-apoptotic factors, such as Bax, to form a complex and then translocate into the mitochondrial membrane [18]. This complex promotes the release of cytochrome C and activates caspase-dependent apoptosis [18]. JNK also regulates FOXO3a activities by affecting MST1 activation [6]. Additional mechanisms governing FOXO3a function by JNK might be related to regulation of Akt or that of some phosphates activities which mediate FOXO3a dephosphorylation [19,20]. However, it is unclear whether JNK is involved in FOXO3a activation in the developing rat brain after HI. Based on previous studies, we hypothesized that the JNK/FOXO3a/Bim pathway is involved in neuronal apoptosis in the developing rat brain after HI. To test this hypothesis, we generated neonatal hypoxia-ischemia brain damage in postnatal day 7 rats to study this pathway in HI-induced neuronal apoptosis.

## Experimental Procedures

### Animal protocols

All animal research was approved by the Sichuan University Committee on Animal Research. Female Sprague–Dawley rats with mixed gender litters were acquired from the animal center of Sichuan University (Chengdu, China). The mother was provided food and water and housed in a temperature- and light-controlled facility until the pups were 7 days old. For the HI model, we used a previously described method [21]. Briefly, each pup was anesthetized with halothane. With the pup supine, the right common carotid artery (CCA) was exposed and permanently ligated with a 7–0 silk suture through a midline cervical incision. After CCA ligation, the pups were returned to the dam for 1 h to recover from anesthesia. A duration of 2.5 h of hypoxia (8% O_2_/92% N_2_) was used to produce the HI injury. Sham controls received halothane anesthesia and exposure of the CCA without hypoxia and ligation of the CCA. The rat brains from sham controls and from 0.5, 6, 24, 48 and 72 h after HI were collected for experiments.

The article "Involvement of the JNK/FOXO3a/Bim Pathway in Neuronal Apoptosis after Hypoxic–Ischemic Brain Damage in Neonatal Rats" was retracted in 2020. Reasons: duplicated images; original data or images not available.

### Intracerebroventricular injection of DMSO and JNK inhibitors

AS601245, a highly specific JNK inhibitor, blocks JNK activity by binding to its ATP-binding site. Pups were anesthetized with 2.5% halothane and intracerebroventricularly infused with vehicle (dimethyl sulfoxide [DMSO], Sigma-Aldrich, USA) or 150 nmol of AS601245 (Alexis Biochemicals, Lausen, Switzerland) dissolved in DMSO into the right cerebral hemisphere 30 minutes prior to HI using a 30-gauge needle with a 5-μL Hamilton syringe (infusion rate 1 μL/min) injections. The AS601245 dose (150 nmol in DMSO) was chosen according to a previous report [22]. The location of each injection was 2 mm rostral, 1.5 mm lateral to bregma, and 2.5 mm deep to the skull surface.

### Fluorescence immunolabeling

To delineate the cellular localization of p-JNK and Bim, double immunolabeling was performed with neuron-specific (NeuN) and astrocytic (GFAP) markers. Paraffin-embedded sections (n = 5) were used for fluorescence double immunolabeling, as described previously [22]. The sections were incubated overnight at 4°C in a mixture of two primary antibodies raised in separate species: rabbit polyclonal antibodies against p-JNK (Thr183/Tyr185; Cell Signaling, 1:100) or Bim (Abcam, 1:200); and mouse monoclonal antibodies against NeuN (Millipore, 1:100) or GFAP (Millipore, 1:100). The sections were then incubated with a 1:80 dilution of a secondary antibody, either FITC- or TRITC-conjugated anti-rabbit or anti-mouse IgG (Sigma Aldrich Inc., USA). The nucleus was stained with 4',6-diamidino-2-phenylindole (DAPI). Images were captured using NIH Image in both the FITC and TRITC channels.

### Western blot analysis

The isolated cortex and hippocampus from the right hemisphere were dissected (n = 5 per group). The samples from the cortex were pooled and processed as described previously [23]. Briefly, cortices were homogenized in ice-cold lysis buffer containing cytosol extraction buffer, consisting of N-[2-hydroxyethyl] piperazine-N′-[2-ethanesulfonic acid] (HEPES; pH 7.9; 10 mmol/L), KCL (10 mmol/L), ethylenediaminetetraacetic acid (EDTA; 0.1 mmol/L), ethylene glycol tetraacetic acid (EGTA; 0.1 mmol/L), dithiothreitol (DTT; 1 mmol/L), phenylmethanesulfonyl fluoride (PMSF; 0.5 mmol/L), the protease inhibitors aprotinin (5 μg/mL) and leupeptin (5 μg/mL), and a phosphokinase inhibitor (10 μg/mL). Lysates were centrifuged at 12,000 g for 30 min at 4°C. Cytosolic and nuclear proteins were purified as described previously followed the Nuclear and Cytoplasmic Extraction Reagents (Pierce, Cat. No.78833). Briefly, cytoplasmic extracts were separated at maximum speed in a microcentrifuge (~16,000 × g) for 5 minutes. Then vortex the insoluble (pellet) fraction and centrifuge the tube at maximum speed (~16,000 × g) in a microcentrifuge for 10 minutes. Protein concentrations were determined using a BCA protein assay kit (Pierce) with bovine serum albumin (BSA) as the standard. Protein samples (100 μg per lane) were separated on 8% SDS-polyacrylamide gels, as described previously [23]. The proteins were then transferred to polyvinylidene fluoride (PVDF) membranes. The membranes were blocked in 5% BSA in TBS containing 0.05% Tween-20 for 1 h at room temperature with rotation. The membranes were incubated for 1 h at room temperature with the following antibodies: rabbit anti-JNK monoclonal antibody (Cell Signaling, 1:1000); rabbit anti-p-JNK (Thr183/Tyr185) polyclonal antibody (Cell Signaling, 1:1000); rabbit anti-Akt polyclonal antibody (Cell Signaling, 1:400); rabbit anti-p-Akt (Ser473) monoclonal antibody (Cell Signaling, 1:400); rabbit anti-FOXO3a polyclonal antibody (Cell Signaling, 1:800); rabbit anti-p-FOXO3a (Ser253) polyclonal antibody (Cell Signaling, 1:800); rabbit anti-Bim polyclonal antibody (Abcam, 1:200); and rabbit anti-CC3 polyclonal antibody (Millipore, 1:100) overnight at 4°C. A rabbit anti-GAPDH polyclonal antibody (Sigma, 1:2000) was used as an internal loading control. The membranes were then incubated with peroxidase-conjugated goat anti-rabbit IgG (Santa Cruz Biotechnology, 1:3000) in blocking solution for 1 h. The signals of the bound antibodies were visualized by enhanced chemiluminescence (Pierce, Rockford, IL). NIH Image was used to quantify the densities of the protein signals on X-ray films after scanning. The protein levels were normalized to GAPDH as a loading control. The relative optical density of the protein bands was measured following subtraction of the film background.

The article "Involvement of the JNK/FOXO3a/Bim Pathway in Neuronal Apoptosis after Hypoxic–Ischemic Brain Damage in Neonatal Rats" was retracted in 2020. Reasons: duplicated images; original data or images not available.

### In vitro kinase assay for JNK

JNK activity was measured using a specific kit (Cell Signaling, USA), and glutathione S-transferase-Jun fusion peptides served as the substrate for JNK, as previously described [22]. In brief, cortex tissue lysates (200 μg) were incubated overnight at 4°C with glutathione S-transferase-Jun fusion protein beads. After washing, the beads were resuspended in kinase buffer containing ATP, and the kinase reaction was allowed to continue for 30 minutes at 30°C. The reactions were halted by adding polyacrylamide gel electrophoresis sample loading buffer. Proteins were separated by electrophoresis on 10% SDS-PAGE, transferred onto PVDF membranes, and incubated with an anti-phospho-c-Jun (Ser63) antibody (Cell Signaling, 1:1000). Immunoreactivity was detected using enhanced chemiluminescence.

### Evaluation of neuropathological injury

Brain injury was evaluated by detecting cell apoptosis as well as calculating infarct volume.

Apoptotic cell death was detected using an In Situ Cell Death Detection Kit (Millipore, Billerica, MA, USA) according to the manufacturer's instructions. Briefly, sections were deparaffinized in xylene, rehydrated through graded ethanol, treated with 0.1 M citrate solution and 3% hydrogen peroxide at room temperature for 10 min and then treated with proteinase K (20 μg/mL) for 7 min. Sections were washed in PBS and incubated at 37°C for 1 h with Fluorescein-FragEL Labeling TdT enzyme. The total cell populations were stained with DAPI. As negative controls, alternate sections were processed in parallel without TdT enzyme.

Brain infarct volume was measured through triphenyltetrazolium chloride (TTC) staining with the method described by Liu et al [24]. Briefly, brains were chilled at −80°C for 4 min. Then five of 2 mm coronal sections were made from the olfactory bulb to the cerebellum and then stained with 1.5% TTC (Sigma, USA) at 37°C for 15 min. After staining, the sections were scanned and measured using image analysis software (NIHimage, USA) to determine the ischemic infarct volume in a blinded manner. Total infarct area was multiplied by the thickness of the brain sections to obtain infarct volume as being previously described [25]. In order to minimize the error introduced by edema, an indirect method for calculating infarct volume was used [26]. The non-infarcted area in the ipsilateral hemisphere was subtracted from that in the contralateral hemisphere, and infarct volume was calculated using the following formula: corrected percentage of infarct volume = (contralateral hemispheric volume-ipsilateral non-infarcted volume) /contralateral hemispheric volume.

### Statistics

The data are represented as the mean±standard deviation (SD). ANOVAs with Bonferroni/Dunnett post hoc tests were performed for multiple comparisons. Significant differences between the two groups were compared using t tests. P<0.05 was considered significant.

The article "Involvement of the JNK/FOXO3a/Bim Pathway in Neuronal Apoptosis after Hypoxic–Ischemic Brain Damage in Neonatal Rats" was retracted in 2020. Reasons: duplicated images; original data or images not available.

## Results

### Expression and distribution of p-JNK and JNK after HI

To quantify p-JNK (active JNK) and total JNK expression after HI in this model, we measured p-JNK and total JNK protein expression levels through Western blot analysis. Total protein was isolated from sham controls as well as from rats at 0.5, 6, 24, 48 and 72 h after HI (each group, n = 5). We found that the total JNK protein was not obviously changed at the different time points compared with sham controls (Fig 1A and 1B). However, p-JNK protein was temporarily reduced at 0.5 h, obviously increased from 6 to 24 h, reached the highest levels at 48 h and remained at a high level at 72 h after HI (Fig 1A and 1B). After normalization to GAPDH, there was a 2.5-fold increase in p-JNK at 48 h after HI compared with sham controls (Fig 1B).

**Fig 1:** Expression and distribution of p-JNK and JNK proteins in the P7 rat brain after HI as detected by Western blot analysis and fluorescence immunolabeling. Samples were obtained from the cortex. Equal levels of protein samples (100 μg) were loaded, and GAPDH served as a loading control. The values are expressed as the relative optical density and represented as the mean±SD (n = 5). Total JNK protein was not obviously changed at different time points compared with sham controls (A). However, p-JNK protein levels transiently decreased at 0.5 h, increased at 6 and 24 h, peaked at 48 h, and lasted until 72 h (A). The JNK and p-JNK expression levels in the HI groups and sham controls were quantified. The data were obtained by densitometry and normalized to GAPDH. *p<0.05, **p<0.01 compared with the sham control (B). (HI, hypoxia-ischemia). The cell type specificity of p-JNK with double fluorescent immunolabeling (n = 5). p-JNK, the neuron-specific marker NeuN and the astrocyte-specific marker GFAP were visualized using a p-JNK antibody followed by a FITC-conjugated secondary antibody (green) and NeuN or GFAP followed by a TRITC-conjugated secondary antibody (red). The nucleus was stained by DAPI (blue). p-JNK (C, D) immunoreactivity colocalized to neurons (yellow) and astrocytes (yellow) in the ischemic cortex. Scale bar, 50 μm.

Because p-JNK is highly expressed at 48 h after HI, double immunofluorescence labeling was performed to determine the cellular localization of p-JNK at 48 h after HI (n = 5). Double staining with the neuronal-specific marker NeuN and the astrocyte-specific marker GFAP showed that p-JNK-immunoreactive cells mainly colocalized with neurons (Fig 1C) and astrocytes (Fig 1D).

### HI promotes FOXO3a dephosphorylation, which induces FOXO3a translocation into the nucleus and upregulates levels of Bim and CC3 proteins

Because FOXO3a has been identified as a principal substrate of JNK in tumor inhibition [5,6], we questioned whether FOXO3a was altered after HI. We quantified both the total FOXO3a and p-FOXO3a protein expression. We found that the total FOXO3a was not markedly changed at the indicated time points (Fig 2A and 2B). However, p-FOXO3a levels decreased from 0.5 to 48 h and returned to baseline at 72 h after HI (Fig 2A and 2B). After normalization to GAPDH, there was an approximately 42% decrease in p-FOXO3a at 48 h after HI compared with the sham controls (Fig 2B). The decrease in p-FOXO3a levels indicates that there was an increase in FOXO3a dephosphorylation.

The article "Involvement of the JNK/FOXO3a/Bim Pathway in Neuronal Apoptosis after Hypoxic–Ischemic Brain Damage in Neonatal Rats" was retracted in 2020. Reasons: duplicated images; original data or images not available.

**Fig 2:** HI promotes FOXO3a dephosphorylation, which induces FOXO3a translocation into the nucleus and upregulates the expression of Bim and CC3. Samples were obtained from the cortex. Equal levels of protein samples (100 μg) were loaded, and GAPDH served as a loading control. The values are expressed as the relative optical density and represented as the mean±SD (n = 5). Total FOXO3a levels remained unchanged at the indicated time points (A). However, p-FOXO3a levels decreased from 0.5 to 48 h and returned to baseline at 72 h after HI (A). Nuclear FOXO3a protein levels obviously increased from 0.5 to 48 h in a time-dependent manner and remained at a high level at 72 h (C). In contrast, the cytoplasmic protein level decreased from 0.5 to 72 h (C). Bim protein was obviously induced at 0.5 h, peaked at 6 h, returned to baseline at 24 h, and then increased again at 48 h and lasted through to 72 h (E). CC3 protein was obviously induced at 6 h, peaked at 24 and 48 h, and remained at a high level at 72 h (E). Total FOXO3a, p-FOXO3a, nuclear and cytosolic proteins of FOXO3a, Bim and CC3 expression in the HI groups and sham controls were quantified. The data were obtained by densitometry and normalized to GAPDH. **p<0.01 compared with the sham control (B, D and F). (HI, hypoxia-ischemia). The cell type specificity of Bim with double fluorescent immunolabeling (n = 5). Bim and the neuronal specific marker NeuN were visualized using an anti-Bim antibody followed by a FITC-conjugated secondary antibody (green) and an anti-NeuN antibody followed by a TRITC-conjugated secondary antibody (red). The nucleus was stained with DAPI (blue). Bim (G) immunoreactivity colocalized to neurons (yellow) in the ischemic cortex. Scale bar, 50 μm.

FOXO3a dephosphorylation has been reported to promote FOXO3a translocation into the nucleus in cultured cerebellar granule neurons deprived of growth factors [12, 13]. We questioned whether HI-induced FOXO3a dephosphorylation would promote FOXO3a translocation into the nucleus. To answer this question, we extracted the nuclear and cytosolic proteins from the cortices and quantified FOXO3a expression separately in the nucleus and cytoplasm using Western blot analysis (Fig 2C). We found that the nuclear protein of FOXO3a obviously increased from 0.5 to 48 h in a time-dependent manner, and it remained at a high level at 72 h (Fig 2C and 2D). After normalization to GAPDH expression, we found that there was an approximately 3.3-fold increase in nuclear protein levels of FOXO3a at 48 h after HI compared with the sham controls (Fig 2D). In contrast, cytoplasmic protein levels evidently decreased from 0.5 to 72 h (Fig 2C and 2D). After normalization to GAPDH expression, there was an approximately 77% decrease in the cytosolic protein levels of FOXO3a at 48 h after HI compared with the sham controls (Fig 2D).

The article "Involvement of the JNK/FOXO3a/Bim Pathway in Neuronal Apoptosis after Hypoxic–Ischemic Brain Damage in Neonatal Rats" was retracted in 2020. Reasons: duplicated images; original data or images not available.

To determine whether Bim, a downstream target gene of FOXO3a, was regulated by FOXO3a translocation into the nucleus, we quantified Bim protein expression using Western blot analysis. We found that Bim protein was obviously induced at 0.5 h, peaked at 6 h, returned to baseline at 24 h, and then increased again at 48 h, which lasted through to 72 h (Fig 2E and 2F). There were approximately 2.4-fold and 1.9-fold increases in Bim expression at 6 and 48 h after HI, respectively, compared with the sham controls (Fig 2F).

Cleaved caspase-3 (CC3) is a key executor of the apoptosis cascade reaction. We quantified CC3 protein expression through Western blot analysis. We found that CC3 protein was obviously induced at 6 h, peaked at 24 and 48 h, and remained at a high level at 72 h (Fig 2E and 2F). There was an approximately 3.7-fold increase in the CC3 protein level at 48 h after HI compared with the sham controls (Fig 2F).

Double immunofluorescence labeling was performed to determine the cellular localization of Bim after HI. Because Bim is highly expressed 48 h after HI, paraffin-embedded sections at 48 h after HI were used (n = 5). As shown in Fig 2, double staining with the neuronal-specific marker NeuN showed that Bim-immunoreactive cells mainly colocalized with neurons in the injured cortices (Fig 2G).

### JNK inhibitor AS601245 rescues the decrease in p-FOXO3a and attenuates FOXO3a translocation into nucleus after HI

To further determine whether JNK was involved in FOXO3a regulation after HI, we utilized AS601245, a highly specific JNK inhibitor, which blocked JNK activity by binding to its ATP binding site [22]. In this study, 150 nM of AS601245 was intracerebroventricularly injected into the injured cerebral hemisphere 30 minutes prior to HI according to a previous report [22]. In vitro kinase assays showed that there was 2.4-fold increase in the levels of phosphorylated GST-c-Jun (p-GST-c-Jun) 48 h after HI compared with sham controls (Fig 3A and 3B), which indicated that HI induced the upregulation of JNK activity. JNK activity was reduced to 41% of the level in the AS601245-treated cortex compared with the DMSO-treated cortex (Fig 3A and 3B), which indicated that JNK activity was blocked by AS601245.

The article "Involvement of the JNK/FOXO3a/Bim Pathway in Neuronal Apoptosis after Hypoxic–Ischemic Brain Damage in Neonatal Rats" was retracted in 2020. Reasons: duplicated images; original data or images not available.

**Fig 3:** JNK inhibitor AS601245 significantly rescued the decrease in p-FOXO3a and attenuated FOXO3a translocation into nucleus after HI with no influence on p-Akt. Samples were obtained from the cortex. A JNK in vitro kinase assay showed a significant increase in phosphorylated GST-c-Jun (p-GST-c-Jun) in the cortex at 48 h after HI compared with sham controls (A). AS601245 pretreatment effectively blocked JNK activity at 48 h after HI compared with the DMSO-treated cortex (A). p-FOXO3a protein levels significantly increased with AS601245 pretreatment at 48 h after HI compared with the DMSO-treated cortex (C). However, total FOXO3a levels remained unchanged (C). Nuclear FOXO3a protein was reduced in the AS601245-treated cortex compared with the DMSO-treated cortex (E). In contrast, the cytosolic protein was increased in the AS601245-treated cortex compared with the DMSO-treated cortex (E). p-Akt and total Akt were not obviously changed at 48 h in the AS601245-treated cortex compared with the DMSO-treated cortex (G). Quantification of total FOXO3a, p-FOXO3a, FOXO3a nuclear, FOXO3a cytoplasmic, total Akt and p-Akt expression in sham controls, HI, DMSO-, and AS601245-treated cortices (D, F, and H). The data were obtained by densitometry and normalized to GAPDH as the loading control. The values are expressed in relative optical density and represented as the mean±SD. For each column, n = 5, *p<0.05, **p<0.01 versus the sham control, #p<0.05, ##p<0.01 compared with DMSO controls (HI, hypoxia-ischemia; AS, AS601245).

We next investigated whether AS601245 pretreatment affected FOXO3a expression and phosphorylation. We found that AS601245 pretreatment significantly increased the expression of p-FOXO3a at 48 h after HI compared with the DMSO controls (Fig 3C and 3D). After normalization to GAPDH, we found that there was approximately a 2.9-fold increase of p-FOXO3a protein at 48 h (Fig 3D). However, total FOXO3a was not markedly changed at 48 h after HI (Fig 3C and 3D).

Because AS601245 pretreatment can rescue the decrease of p-FOXO3a after HI, we further investigated whether JNK was involved in the regulation of FOXO3a translocation from the cytoplasm to the nucleus. We found that FOXO3a was upregulated in the nucleus but downregulated in the cytoplasm 48 h after HI (Fig 3E and 3F). However, AS601245 treatment obviously reduced the FOXO3a nuclear protein and increased the FOXO3a cytosolic protein compared with the DMSO-treated cortex (Fig 3E and 3F). After normalization to GAPDH expression, we found that AS601245 blocked approximately 58% of the FOXO3a nuclear protein (Fig 3F). Meanwhile, there was an approximately 2.9-fold increase in FOXO3a cytosolic protein at 48 h after HI (Fig 3F) in the AS601245-treated cortex compared with the DMSO-treated cortex.

The article "Involvement of the JNK/FOXO3a/Bim Pathway in Neuronal Apoptosis after Hypoxic–Ischemic Brain Damage in Neonatal Rats" was retracted in 2020. Reasons: duplicated images; original data or images not available.

There is crosstalk between the pro-apoptotic JNK pathway and the pro-survival Akt pathway at multiple levels [27,28]. To further investigate whether the regulation of FOXO3a by JNK after HI is related to Akt, we examined the expression of p-Akt and Akt protein after JNK was blocked with AS601245 using Western blot analysis. We found that both the p-Akt and total Akt levels were not changed at 48 h in the AS601245-treated cortex compared with the DMSO-treated cortex (Fig 3G and 3H), suggesting that the regulation of FOXO3a by JNK is independent of Akt in this study.

### JNK inhibitor AS601245 decreases levels of Bim and CC3 proteins and reduces brain damage after HI

To further understand whether JNK inhibition could regulate a pro-apoptotic protein Bim, one of the FOXO3a target genes, and CC3 in this model, we used Western blot assays to detect the expression of Bim and CC3 protein after JNK was blocked with AS601245. We found that the Bim and CC3 protein levels were significantly reduced at 48 h in the AS601245-treated cortex compared with the DMSO-treated cortex (Fig 4A and 4B). After normalization to GAPDH expression, we found that there was approximately a 43% decrease in Bim protein levels at 48 h (Fig 4B) and approximately a 61% decrease in CC3 protein levels at 48 h (Fig 4B) in the AS601245-treated cortex compared with the DMSO-treated cortex.

**Fig 4:** JNK inhibitor AS601245 decreased levels of Bim and CC3 proteins and reduced neuronal apoptosis and brain infarct volume in P7 rat after HI. Samples were obtained from the cortex. Bim and CC3 protein levels were significantly reduced at 48 h in the AS601245-treated cortex compared with the DMSO-treated cortex (A). Cell apoptosis was detected by TUNEL staining with the In Situ Cell Death Detection Kit (Merck Millipore) according to the manufacturer's protocol. Ten fields were chosen randomly at 400x magnification to count the apoptotic and total cells. The apoptotic index (AI) was calculated as follows: AI = (number of apoptotic cells/total number counted) ×100%. TUNEL-positive cells were not detected in the sham controls (C). However, the positive cells were increased at 6 h (data not shown) and 24 h (data not shown) and peaked at 48 h (D) after HI. Meanwhile, AS601245 pretreatment obviously reduced cellular apoptosis at 48 h after HI (F) and decreased the infarct volume 7 days after HI significantly (Fig 4H), compared with the DMSO controls (Fig 4E and 4H,). The cell apoptosis index in the AS601245-treated brain cortex was decreased by 59% compared with the DMSO-treated brain cortex (Fig 4G). The infarct volume in the AS601245-treated brain was decreased by 58% compared with the DMSO controls (Fig 4I).

The article "Involvement of the JNK/FOXO3a/Bim Pathway in Neuronal Apoptosis after Hypoxic–Ischemic Brain Damage in Neonatal Rats" was retracted in 2020. Reasons: duplicated images; original data or images not available.

Because the blockade of JNK activity by AS601245 decreased the expression of Bim and CC3, we investigated whether cellular apoptosis could be blocked by the downregulation of Bim and CC3. Brain sections from sham controls and 0.5, 6, 24, 48 and 72 h after HI as well as from AS601245-treated sections were examined for cellular apoptosis using TUNEL staining (each group, n = 5). We found that TUNEL-positive cells were not detected in the sham controls (Fig 4C) as well as at 0.5 h (data not shown) after HI. However, the number of positive cells increased at 6 h (data not shown) and 24 h (data not shown) and peaked at 48 h (Fig 4D) after HI. Meanwhile, we found that AS601245 pretreatment obviously reduced cellular apoptosis at 48 h after HI (Fig 4F), and decreased the infarct volume 7 days after HI significantly (Fig 4H), compared with the DMSO controls (Fig 4E and 4H,). The cell apoptosis index in the AS601245-treated brain cortex was decreased by 59% compared with the DMSO-treated brain cortex (Fig 4G). The infarct volume in the AS601245-treated brain was decreased by 58% compared with the DMSO controls (Fig 4I).

## Discussion

In this study, we first showed that the JNK/FOXO3a/Bim pathway was involved in neuronal apoptosis in the developing rat brain after HI. First, we found that JNK phosphorylation and the reduction of p-FOXO3a preceded neuronal apoptosis, suggesting that JNK phosphorylation and FOXO3a dephosphorylation were involved in mediating HI-induced brain damage. Second, FOXO3a dephosphorylation induced FOXO3a translocation from the cytoplasm into the nucleus, which upregulated levels of pro-apoptosis proteins, such as Bim and CC3. Third, pretreatment with AS601245, a highly specific JNK inhibitor, clearly increased FOXO3a phosphorylation, leading to a decrease in FOXO3a translocation from the cytoplasm to the nucleus and levels of Bim and CC3 proteins. Finally, JNK inhibition with AS601245 reduced neuronal apoptosis and brain infarct volume after HI.

JNK is an important stress-responsive kinase that is activated by various forms of brain insults. The activated form of JNK is p-JNK. After phosphorylation, activated JNK can activate its downstream transcriptional factors, triggering the expression of pro-apoptotic target gene Bim, and inducing cell apoptosis [4]. In addition to Bim, JNK is involved in regulation of 14-3-3 protein phosphorylation [3]. Serine phosphorylation of 14-3-3 protein promotes translocation of Bax to mitochondria that is essential process to initiate mitochondrial apoptosis [3]. Using double immunofluorescence labeling, we found that p-JNK (active JNK) was mainly expressed in the neurons and astrocytes in the injured cortex (Fig 1C and 1D). The levels of p-JNK decreased temporarily at 0.5 h and obviously increased from 6 to 72 h after HI (Fig 1A and 1B), indicating that HI facilitated JNK phosphorylation and increased its activity. Our findings are in accordance with previous reports [29]. Although there are contradicting reports that p-JNK increases at 0.5 h after global ischemia in an adult rat model [3], we believe that these discrepancies may be due to differences in the animal age and the ischemic model.

The article "Involvement of the JNK/FOXO3a/Bim Pathway in Neuronal Apoptosis after Hypoxic–Ischemic Brain Damage in Neonatal Rats" was retracted in 2020. Reasons: duplicated images; original data or images not available.

Previous studies have revealed that JNK regulates the FOXO3a activity at different levels and in multiple modes [14,15]. Phosphorylation/dephosphorylation play a key role in the regulation of FOXO3a subcellular localization and transcriptional activities [11]. Acetylation of FOXO proteins has been described as important for their activity as well. Acetylation of FOXO proteins by acetylases such as CBP and p300 inhibits their activity and increases the response of them to oxidative stress [9]. JNK also regulates FOXO3a activities by effecting MST1 activation [6]. We found that p-FOXO3a decreased at 0.5 h and was maintained at a low level at 48 h after HI (Fig 2A and 2B). Because p-FOXO3a, the inactive form of FOXO3a, decreased and the total FOXO3a level was not changed, dephosphorylated FOXO3a, the active form of FOXO3a, increased. Once FOXO3a dephosphorylation occurs, FOXO3a translocation from the cytoplasm into the nucleus is facilitated [12,13]. We found that translocation of FOXO3a into the nucleus occurred along with the reduction in the expression of p-FOXO3a at 0.5 h after HI (Fig 2C and 2D). Meanwhile, the expression of the pro-apoptotic protein Bim increased and peaked at 6 h after HI (Fig 2E and 2F), which was earlier than the peak time for neuronal apoptosis (Fig 4D). The expression of CC3 peaked at 24 and 48 h, which was in accordance with the peak time for the neuronal apoptosis. (Fig 2E, Fig 4D). These findings demonstrated that the reduction of p-FOXO3a promoted the translocation of FOXO3a into the nucleus and induced the expression of the pro-apoptotic proteins Bim and CC3, leading to neuronal apoptosis after HI. We also found that Bim expression was not entirely in accordance with the nuclear translocation of FOXO3a at 24 h after HI because nuclear FOXO3a protein remained at a high level, whereas Bim protein levels returned to baseline. One possible reason for this discrepancy may be due to the degradation of Bim by the ubiquitin-proteasome pathway as previously reported [30].

The article "Involvement of the JNK/FOXO3a/Bim Pathway in Neuronal Apoptosis after Hypoxic–Ischemic Brain Damage in Neonatal Rats" was retracted in 2020. Reasons: duplicated images; original data or images not available.

Contrary to the pro-apoptotic JNK pathway, Akt inhibits cellular apoptosis through the negative regulation of FOXO3a activities [12,31]. There is crosstalk between the pro-apoptotic JNK pathway and pro-survival Akt pathway at multiple layers and levels [27, 28]. In this study, the phosphorylation of JNK after HI occurred along with the reduced expression of p-FOXO3a and the translocation of FOXO3a into the nucleus. Therefore, we wished to determine whether JNK participates in the regulation of FOXO3a-mediated neuronal apoptosis. We injected the JNK-specific inhibitor AS601245 into the rat brain 30 minutes prior to HI. AS601245 protects neurons from injury in the adult global ischemic model, neonatal hypoxia-ischemia brain damage (HIBD) model and white matter injury model [22,32,33]. Toxicological studies have shown that AS601245 exerts no influence on physiological indexes, such as arterial blood pressure, blood sugar, body temperature, etc. [32]. In this study, JNK activity in the AS601245-treated cortex was reduced to 41% of the level compared to the DMSO-treated cortex (Fig 3A and 3B), indicating that JNK activity was blocked by AS601245. Meanwhile, we found that AS601245 treatment obviously increased p-FOXO3a expression (Fig 3C and 3D), which significantly attenuated FOXO3a in the nucleus but increased its level in the cytoplasm (Fig 3E and 3F). These findings suggested that AS601245 reduced FOXO3a translocation from the cytoplasm to the nucleus. The reduction of FOXO3a translocation by JNK inhibition might be mediated via increased p-FOXO3a.

Because FOXO3a is downstream of Akt [12], we questioned whether Akt is involved in the regulation of JNK/FOXO3a. Surprisingly, we found that JNK inhibition by AS601245 did not affect the level of p-Akt after HI (Fig 3G and 3H). This finding suggests that the regulation of FOXO3a phosphorylation and its translocation into the nucleus by the JNK signal pathway was not mediated by Akt. The mechanism by which JNK regulates FOXO3a in an Akt-independent manner after HI is not clear. JNK-regulated phosphatase activities may be involved in the dephosphorylation of FOXO3a [19,20].

The transcription factor FOXO3a can activate Bim gene expression and promote caspase-independent apoptosis [13]. In addition, the direct effect of JNK on Bim and consequent Bax translocation to mitochondria are also essential processes to initiate mitochondrial apoptosis [3]. We further studied whether the inhibition of JNK by AS601245 could downregulate the expression of Bim and CC3 and decrease cellular apoptosis. We found that AS601245 not only obviously reduced the expression of Bim and CC3 (Fig 4A and 4B), it also significantly inhibited neuronal apoptosis and reduced brain infarct volume after HI (Fig 4F and 4H). Our findings are consistent with a recent report that showed JNK inhibition may provide neuroprotection by downregulating Bim after adult ischemic brain injury [3].

The article "Involvement of the JNK/FOXO3a/Bim Pathway in Neuronal Apoptosis after Hypoxic–Ischemic Brain Damage in Neonatal Rats" was retracted in 2020. Reasons: duplicated images; original data or images not available.

In summary, we have shown that the JNK/FOXO3a/Bim pathway is involved in neuronal apoptosis in the developing rat brain after HI, and JNK’s regulation of FOXO3a may be independent of Akt. Agents targeting JNK might provide insight into the protective mechanisms involved in neonatal HI.
